# Nanomedicines Targeting Metabolism in the Tumor Microenvironment

**DOI:** 10.3389/fbioe.2022.943906

**Published:** 2022-08-05

**Authors:** Mengdi Ren, Xiaoqiang Zheng, Huan Gao, Aimin Jiang, Yu Yao, Wangxiao He

**Affiliations:** ^1^ Department of Oncology, The First Affiliated Hospital of Xi’an Jiaotong University, Xi’an, China; ^2^ Institute for Stem Cell and Regenerative Medicine, The Second Affiliated Hospital of Xi’an Jiaotong University, Xi’an, China; ^3^ Department of Talent Highland, The First Affiliated Hospital of Xi’an Jiaotong University, Xi’an, China

**Keywords:** metabolic reprograming, tumor microenvironment, nanomedicine, metabolism, cancer treatment

## Abstract

Cancer cells reprogram their metabolism to meet their growing demand for bioenergy and biosynthesis. The metabolic profile of cancer cells usually includes dysregulation of main nutritional metabolic pathways and the production of metabolites, which leads to a tumor microenvironment (TME) having the characteristics of acidity, hypoxic, and/or nutrient depletion. Therapies targeting metabolism have become an active and revolutionary research topic for anti-cancer drug development. The differential metabolic vulnerabilities between tumor cells and other cells within TME provide nanotechnology a therapeutic window of anti-cancer. In this review, we present the metabolic characteristics of intrinsic cancer cells and TME and summarize representative strategies of nanoparticles in metabolism-regulating anti-cancer therapy. Then, we put forward the challenges and opportunities of using nanoparticles in this emerging field.

## Introduction

Metabolic reprogramming, a hallmark of cancer, is considered to be one of their driving forces. It endows cancer cells with the potential for initiation and proliferation in the nutrient-deficient tumor microenvironment (TME) (Yoshida, 2015; Martínez-Reyes and Chandel, 2021). Cancer cells usually abandon the efficient metabolic pathway used by most normal cells and switch to alternative pathways that produce less energy and more materials to meet the needs of biosynthesis and bioenergy synthesis (Vander Heiden et al., 2009). The metabolic reprogramming is regulated by an oncogene and influenced by an external TME. For example, the metabolic composition of the TME can affect the metabolic phenotype of cancer cells (Seth Nanda et al., 2020). Other cells within TME, including stromal and immune cells, form a metabolic network and crosstalk to regulate tumor growth and anti-cancer immunity (Guo et al., 2019; Pacella and Piconese, 2019; Vettore et al., 2020). Changes in the cellular metabolism of these cells also involve nutrient limitation and immunosuppressive functions (Yin et al., 2019). Moreover, various metabolites within TME play an important role in cancer cell behavior and cellular communication (Sola-Penna et al., 2020). Thus, the metabolism of various cells and metabolites in TME plays pivotal roles in tumor progression and maintenance.

As metabolism is the basic determinant of the viability and function of cancer and noncancer cells in TME (10), targeting metabolic pathways opens up a new way to thwart tumor growth (Elia and Haigis, 2021). However, therapeutic progress in disrupting cancer metabolism is limited (Stine et al., 2022). A part of the reason is that cellular metabolism is huge and complex networks of enzymes and compounds acting together. The technical limitations also make all elements still not fully understood. Another part is that strategies for targeting the intrinsic metabolism of cancer cells usually do not consider the metabolism and crosstalk of noncancer cells within TME (Stine et al., 2021). This means that blocking only one metabolic pathway may be counterproductive because many pathways of cancer cells are also important for immune cells.

Over the past few decades, nanotechnology has made brilliant achievements in diagnosis, imaging, and cancer treatment *in vivo* (Liu et al., 2019; Yang et al., 2020a; Irvine and Dane, 2020). Because of various unique advantages of nanomedicine, such as good biocompatibility, biological degradation, high targetability, and therapeutic efficacy, the development of nanotechnology is leading anti-cancer therapy into a new era for multimode treatment (Yan et al., 2019; Yan et al., 2020a; Li et al., 2021a; Yan et al., 2022), including targeting metabolism in tumors. The strategy of using nanomedicines to modulate metabolic pathways offers a promising opportunity to fight against tumors. Nanomedicine can specifically target cancer cells by regulating their physicochemical properties, thereby controlling the pharmacokinetics and biodistribution of compounds (Wicki et al., 2015; Li et al., 2021b; Liu et al., 2022). Nanomedicine can also be used as carriers carrying multiple therapeutic cargos capable of metabolic modulation or acting with metabolites in TME to improve immunosuppressive TME [(Cao et al., 2021); (Yan et al., 2021a)], which results in more effective and less toxic effects (Yang et al., 2019; She et al., 2020; Zheng et al., 2021).

In this review, we will briefly summarize the representative work of nanoparticles contributing to the metabolic modulation in the context of cancer (Table 1) and TME (Table 2). In addition, we will discuss and analyze some possible reasons limiting the applications and prospect new insights into this field.

**TABLE 1:** Representative nanoparticles targeting cancer metabolism.

Metabolism Pathway	Nanoparticle	Nanocarrier Material	Size	Cargo	Targets	Mechanism	Indication	Advantages	References
Aerobic glycolysis	Nanoenabled Energy Interrupter	ZIF‐8; hydrophilic shell	117 nm	GLUT1 mRNA‐cleaving DNAzyme	GLUT1 mRNA	GLUT1 specific depletion	glycolysis Inhibition therapy	HAase‐responsive and pH‐sensitive; cut off glucose supply	Wu et al. (2022)
	GNR/HA-DC	plasmonic gold nanorods	768 nm	HA-targeting moiety and DC	GLUT1	inhibiting glucose uptake and glycolysis	improved PTT	HAase‐responsive; overcoming the heat endurance of tumor cells	Chen et al. (2017a)
	l-Arg-HMON-GOx	hollow mesoporous organosilica nanoparticle	pore size of 3.7 nm	Gox and l-Arg	endogenous glucose	cutting off the energy supply and generating toxic H2O2	synergistic cancer starving-like/gas therapy	Glucose-Responsive; without the need for external excitation	Fan et al. (2017)
	Lip-(2DG + Dox)	liposomes	<200 nm	Dox and 2DG	hexokinase	inhibit glycolysis; promote mitochondrial depolarization and apoptosis	tumor-specific chemotherapy	mitigates the harmful side effect of chemotherapy	Yang et al. (2020b)
	2DG-PLGA-NPs	poly (lactic-co-glycolic acid) nanoparticles	120 nm	2DG	hexokinase	induce antitumor immunity	overcome the immune-resistance	decreasing lactate production and increasing T cells in tumors	Sasaki et al. (2021)
	GSH-responsive nanoprodrug	pluronic F126	100 nm	LND and NLG919	HK II and IDO-1	restrained glycolysis and reduce the kynurenine	alleviate immunosuppression	GSH-Responsive; destructed the immunosuppressive microenvironment	Liu et al. (2021)
	RBCm@Ag-MOFs/PFK15 (A-RAMP)	metal–organic frameworks; red blood cell membrane shell	20 nm	PFK15	PFK-2/FBPase-2/PFKFB	inhibit glycolysis	targeted B-cell lymphoma	CD20 aptamer-targeting	Zhao et al. (2020a)
Mitochondrial respiration	Copper-depleting nanoparticle (CDN)	semiconducting polymer nanoparticle	86.6/81 nm	CDM and SPN	mitochondrial ETC	shifts metabolism pattern	treat TNBC	specific accumulation to be less toxic	Cui et al. (2021)
	polymersome nanoparticle	amphiphilic grafted-polyphosphazene nanovesicle	135.9 nm	VES and DOX·HCl	mitochondrial ETC	inducing mitochondrial malfunction and apoptosis	overcome multidrug resistance	result in mitochondria dysfunctions	Liang et al. (2021)
	IR780@Pt NPs	β-CD and adamantyl group	150 nm	Pt-CD and IR780	mitochondrial	mitochondrial dysfunction	chemotherapy synergetic treatments	track tumor accumulation; guide the NIR laser irradiation	Zhang et al. (2021b)
	UCNPs- MSN- MnO2 (UNMM)	the mesoporous silicon middle layer; MnO2 gatekeeper layer	36 nm	MnO2, Ce6, and ATO	mitochondrial ETC	inhibit respiration metabolism and generate O2	enhanced PDT	inhibiting oxygen metabolism and generating oxygen	Wang et al. (2020a)
	VSeM-N=CH-PEG	acidity-cleavable PEG	∼100 nm	VES and MTX	mitochondrial ETC	interfere ETC	synergistic oxidation-chemotherapy	self-targeting activation and ROS regeneration	Li et al. (2020a)
	ACSN	carrier-free	193.5 nm	ATO and Ce6	mitochondrial ETC	interrupt ETC, relieve the hypoxia microenvironment	improving PDT	self-delivery; reverse the tumor hypoxia	Zhao et al. (2020b)
Glycolysis and mitochondrial metabolism	LMGC	liquid metal nanoparticles	250 nm	Gox	endogenous glucose	inhibit glycolysis; increased H2O2 level	synergetic PTT	acidity-responsive; reduce heat resistance	Ding et al. (2022)
Glutamine metabolism	Pt-Pd@DON	porous Pt–Pd nanoflowers	97 nm	DON	binds covalently to multiple enzymes that use glutamine	glutamine analog	electrodynamic synergetic treatments	motivate the protective immune response	Chen et al. (2022)
	ABFP NPs	BSA-based NPs	140 nm	purpurin	GDH1	inhibiting the decomposition of mitochondrial Gln	synergetic chemodynamic treatments	real-time tracking of the Fenton reaction	Xu et al. (2021)
GSH depeltion	AM-L@NBS	DSPE-PEG2k-Maleimide; CD44-specific polypeptide (A6) modified liposome	60–80 nm	maleimide	GSH	exhaust intracellular GSH; upregulate ROS levels	amplify PDT	CD44-specific targeting; good specificity and biocompatibility	Shi et al. (2021)
	CuO2@mPDA/DOX-HA (CPPDH)	copper peroxide	106 nm	HA; PA; DOX	GSH	Cu + catalyzed H2O2 to produce •OH	synergetic PDT/CDT	HA-targeting and acidic-triggering	Xiao et al. (2021)

NPs, nanoparticles; HA, hyaluronic acid; DC, diclofenac; GOx, glucose oxidase; 2DG, 2-Deoxy-d-glucose; PLGA, poly (lactic-co-glycolic acid); LND, lonidamine; HK II, hexokinase II; IDO-1, 2,3-dioxygenase 1; A-RAMP, RBCm@Ag-MOFs/PFK15; PFK15, 1-(4-pyridyl)-3-(2-quinoline)-2-propyl-1-one; PFKFB3, 6-phosphofructo-2-kinase/fructose-2, 6-bisphosphatase 3; CDN, Copper-depleting nanoparticle; CDM, copper-depleting moiety; SPN, semiconducting polymer; ETC, electron transport chain; VES, vitamin E succinate; DOX·HCl, Doxorubicin hydrochloride; β-CD, β-cyclodextrin; CDDP, cisplatin; UNMM, UCNPs- MSN- MnO2 nanocomposites; Ce6, chlorine 6; ATO, atovaquone; MTX, methotrexate; PDT, photodynamic therapy; PTT, photothermal therapy; DON, 6-diazo-5-oxo-l-norleucine; GDH1, Glutamate dehydrogenase 1; CDT, chemodynamic therapy; CPPDH, CuO2@mPDA/DOX-HA; PA, photoacoustic; and DOX, doxorubicin.

**TABLE 2:** Representative nanoparticles targeting TME metabolism.

Metabolism pathway	Name	Nanocarrier material	Size	Cargo	Targets	Mechanism	Indication	Advantages	References
Lactic acid	PMLR	mRBC-camouflaged hollow MnO2 catalytic nanosystem	65 nm	3PO and LOX	lactic acid oxidation and glycolysis	catalyze the oxidation reaction of lactic acid and inhibit glycolysis	synergistic metabolic therapy and immunotherapy	remove lactic acid; lead to an immunocompetent TME	Gao et al. (2019b)
Lactic acid	PFOB@TA-Fe (III)-LOX, PTFL	TA-Fe (III) coordination complexes-coated PFOB	182 ± 13 nm	LOX	lactic acid oxidation	dual-depletion of lactate and ATP with hydroxyl • OH radicals’ generation	cascade metabolic-CDT	provide imaging guidance	Tian et al. (2021)
Kynurenine	1-MT@i-aCMP nanosheets	aCMP nanosheets	200 ± 18 nm	IDO inhibitors	IDO-1	IDO inhibition; evokes ICD by generating ROS and hyperthermia under NIR irradiation	reversing Immunosuppression in hypoxic and immune-cold tumors	reshaped cold tumors into hot ones	Jiang et al. (2021)
Kynurenine	AIM NPs	CaCO3	174.2 nm	4PI	IDO-1	suppress Kyn accumulation	reinforces radiotherapy by reprogramming the immunosuppressive metabolic microenvironment	pH-responsive; suppress the distant tumors; result in immune memory responses	Wang et al. (2022b)
Prostaglandin E2 (PGE2)	Cele-BMS-NPs	human serum albumin	43.5 ± 4.0 nm	BMS-202; GSH-activatable prodrug of celecoxib	COX-2	inactivating COX-2	regulate immunosuppressive pivot	pH-sensitive; resolve the different pharmacokinetic profiles and the spatial obstacles	Feng et al. (2022)
Hypoxia and kynurenine	PF-PEG@Ce6@NLG 919 NPs	fluorinated polymeric	94.6 nm	Ce6 and NLG919	IDO-1; Hypoxia	the combined action of hypoxia alleviation-induced PDT and IDO inhibitor	hypoxia alleviation-triggered enhanced photodynamic therapy	hypoxia alleviation-triggered	Xing et al. (2019)
Lipid metabolism	aCD3/F/AN	F/Ans	∼150 nm	fenofibrate	activate T cells	activate fatty acid metabolism; restore mitochondrial functions	immunometabolism therapy	enhances the production of various cytokines in tumor tissues	Kim et al. (2021)
Lipid metabolism	T-Tre/BCN-Lipo-Ava	liposomes	91.5 nm	Ava	increase the concentration of cholesterol in the T cell membrane	induced rapid T cell receptor clustering and sustained T cell activation	cell-surface anchor-engineered T cells	safe cell-surface anchor-engineered T cells	Hao et al. (2020)

RBC, red blood cell membrane; 3PO, 3-(3-pyridinyl)-1-(4-pyridinyl)-2-propen-1-one; LOX, lactate oxidase; CDT, chemodynamic therapy; IDO-1, 2,3-dioxygenase 1; AIM NPs, acidity-IDO1-modulation nanoparticles; CaCO3, carbonate; 4PI, 4-phenylimidazole; Kyn, kynurenine; PGE2, Prostaglandin E2; GSH, glutathione; COX-2, cyclooxygenase-2; Ce6, Chlorin e6; F/Ans, amphiphilic poly (γ-glutamic acid)-based nanoparticles; and Ava, Avasimibe.

## Cancer Cell Metabolism and Targets

To meet the demands of unrestrained proliferation, cancer cells undergo specialized alterations in various metabolic pathways (DeBerardinis and Chandel, 2016). In general, the characteristics of cancer cells metabolically reprogramming mainly involves the abnormality of the main nutritional metabolic pathways (glucose, amino acid, and lipids) (Guo et al., 2019).

In both normal and cancerous cells, glucose is the source of energy via glycolysis in the cytoplasm and oxidative phosphorylation (OXPHOS) in the mitochondrion. The pentose phosphate pathway (PPP), a vital branch of glycolysis, makes an important contribution to helping cancerous cells meet the needs of anabolism and anti-oxidative stress (Patra and Hay, 2014). Glucose breakdown generates pyruvic acid providing acetyl-CoA for the tricarboxylic acid (TCA) cycle, which is a hub of bioenergy synthesis and precursor for biosynthesis (Eniafe and Jiang, 2021). The uptake and upregulated *de novo* synthesis of amino acids is also abnormally upregulated, which has diverse and important roles in tumors (Lukey et al., 2017). The enhancement of glutamine metabolism is the main feature that promotes tumor progression by facilitating energic synthesis and biosynthesis (Yoo et al., 2020). Amino acid metabolism also includes pathways of one-carbon metabolism, TCA cycle, and reduced glutathione synthesis (Wei et al., 2020). In addition, cancer cells show an increase in exogenous lipids uptake and hyperactivating lipogenesis pathway to produce key lipid cell structures, such as cell membranes. Fatty acids (FAs) and cholesterol are synthesized from glucose-derived cytoplasmic acetyl-CoA. Long-chain fatty acids split into acetyl-CoA via fatty acid β oxidation (FAO) to drive the TCA cycle in order to produce adenosine triphosphate (ATP) and biosynthesis, which is also important for proliferation, drug resistance, and metastatic progression in cancer (Ma et al., 2018). In this section, we briefly present the fundamental targets of metabolism in cancer cells and mainly focus on recent nanoparticle efforts to target cancer metabolism (Figure 1).

**FIGURE 1:** The metabolism of cancer cells. Enhanced aerobic glycolysis, also known as the Warburg effect, enables cancer cells to generate large amounts of biomolecules for biomass production. Glutamine is converted into glutamate and ammonia in the process of glutaminolysis. The upregulation of *de novo* lipid synthesis and fatty acid oxidation is related to bioenergy synthesis and signaling molecules needed for proliferation. Various nanomedicines can target these metabolic vulnerabilities in cancer cells and improve therapeutic effects, including photothermal, gene, chemo-, and immunotherapy. ETC, electron transport chain; OXPHOS, oxidative phosphorylation; and TCA, tricarboxylic acid cycle.

### Aerobic Glycolysis and Mitochondrial Aerobic Respiration

Glucose is the main source of energy available to all cells. The utilization of glucose starts from the uptake by cells and conversion to glucose 6-phosphate, which could enter into glycolysis to yield pyruvate, glycogen synthesis, and the PPP. The breakdown of energy sources includes glycolysis, the TCA cycle, and oxidative phosphorylation OXPHOS (36). Under aerobic conditions, normal cells mainly produce energy through the OXPHOS pathway, and glycolysis is inhibited, while tumor cells, even under aerobic conditions, mainly produce ATP through glycolysis, which is called aerobic glycolysis, namely, the Warburg effect (Warburg, 1925; Kuntz et al., 2017; Courtney et al., 2018). Metabolic targeting therapy of tumor glucose metabolism is the most common anti-cancer nanoparticle strategy, which mainly focuses on glycolysis and mitochondrial OXPHOS.

Glucose is an object that can be controlled directly. Extracellular glucose is transported into the cell through glucose transporters (GLUTs), which makes it a potential therapeutic target for suppressing tumors (Zhang et al., 2021a). A novel paradigm therapy of systematic energy exhaustion is proposed to synergize the glycolysis inhibition and GLUT1 depletion using a “nano‐enabled energy interrupter,” which enables energy exhaustion via zinc (II) interference for effective tumor therapy (Wu et al., 2022). Chen et al. (2017a) prepared a nanodrug GNR/HA-DC, which contains hyaluronic acid (HA)-targeting part and diclofenac (DC, a GLUT1 inhibitor). Upon specifically targeting CD44, the GNR/HA-DC shows that it can sensitize tumor cells for photothermal therapy (PTT) by inhibiting anaerobic glycolysis. Besides, glucose is catalyzed by glucose oxidase (GOx), which could help convert glucose into gluconic acid and toxic H2O2, thereby inhibiting the process of glycolysis and enhancing tumor therapy (Fan et al., 2017; Ding et al., 2022). A multifunctional liquid metal-based nanoparticle attached with GOx and mineralizing calcium carbonate can inhibit glycolysis and mitochondrial metabolism to improve PTT efficiency (Ding et al., 2022). Another report of nanoparticles, as a biocompatible nanocarrier, is used to deliver GOx, which also yields a significant anti-cancer effect (Fan et al., 2017).

Other candidate approaches include the targeting of metabolites in glycolysis or inhibition of key enzymes. Key enzymes include hexokinase (HK), phosphofructokinase (PFK), and pyruvate kinase (such as M-type isozyme, PKM). (DiTullio and Dell’Angelica, 2019) 2-Deoxy-D-glucose (2DG) is a glucose analog (Ralser et al., 2008), which can inhibit HK and prevent glycolysis. Synthesized a liposome nanoparticle that is co-loaded with doxorubicin (Dox) and 2DG in liposomes could inhibit glycolysis of cancerous cells, which also leads to mitochondrial depolarization and subsequent apoptosis Yang et al. (2020b). Sasaki et al. (2021) also developed 2DG-encapsulated poly (lactic-co-glycolic acid) (PLGA) NPs, which shows antitumor immunity and cytotoxicity in tumors. As an effective inhibitor of glycolysis, Lonidamine (LND) is an effective inhibitor of hexokinase II (HK II), a rate-limiting enzyme for glycolysis pathways. A GSH-responsive nanodrug that is loaded with LND restrains the glycolysis of tumor cells and inhibits tumor growth (Liu et al., 2021). In a similar manner, a nanodrug consists of 1-(4-pyridyl)-3-(2-quinoline)-2-propyl-1-one (PFK15), which is a PFKFB3 inhibitor targeting glycolysis metabolism (Zhao et al., 2020a). This work shows that synchronously molecular-targeting and metabolic-regulating can exert a better anti-tumor effect.

However, cancer cells not only metabolize glucose by glycolysis but also produce ATP via mitochondrial glucose metabolism (Weinberg and Chandel, 2015). This hybrid energetic metabolic pattern makes the traditional single metabolic anti-cancer therapy hardly obtain satisfactory efficacy (Gottschalk et al., 2004). For example, triple-negative breast cancer (TNBC) is insensitive to enzyme inhibitors targeting glucose transport, which makes OXPHOS a more important target for the treatment of TNBC (52). Therefore, Cui developed a mitochondria-targeted, copper-depleting nanoparticle, which is effective against TNBC that depends on oxidative phosphorylation (Koppenol et al., 2011). This nanoplatform has a positive surface charge, which helps accumulation in the mitochondria and local depletion of copper. However, cancer cells will compensate by increasing the other pathway to produce ATP if a single pathway of glucose metabolism is inhibited (Gottschalk et al., 2004). Therefore, many energy-depletion strategies of nanoparticles are designed to block both energy synthesis pathways synergistically (Ding et al., 2022; Dong et al., 2022). A cancer cell membrane camouflaged nanoinhibitor co-encapsulates OXPHOS inhibitor and glycolysis inhibitor for synergistically blocking two pathways that significantly suppress tumor growth (Dong et al., 2022), while some studies have confirmed that the strategy of targeting mitochondria can also reduce the occurrence and metastasis of tumors (Zhang et al., 2021b; Lin et al., 2021). The common scheme is inhibiting mitochondrial complexes of the electron transport chain (ETC). Vitamin E succinate (VES) is a molecule that can bind with the ubiquinone in Complex II to interfere with the mitochondrial respiratory metabolism (Dong et al., 2011). Inducing mitochondrial malfunction through VES loaded in a self-assembly polymersome nanoplatform is an appealing strategy to improve cancer therapy and overcome multidrug resistance (Liang et al., 2021). A pH/ROS cascade-responsive vitamin E nanodrug releases VES interfering with the ETC to aggravate tumor cell killing (Li et al., 2020a). Atovaquone (ATO) is an ETC inhibitor that disturbs the activity of OXPHOS, which is another commonly nanoloaded drug (Xia et al., 2019). A carrier-free self-delivery nanomedicine based on photosensitizer (PSs) Ce6 and OXPHOS inhibitors of ATO exhibited marked efficacy and low toxicity (Zhao et al., 2020b). An intelligent multilayer nanostructure was also designed based on ATO (61): the decomposition of outer MnO2 can create O2, which elevates the oxygen content of TME. Then, the released ATO molecules of the middle mesoporous silicon layer could effectively inhibit tumor respiration metabolism.

As glucose metabolism is a crucial regulatory target in tumors, its regulation has attracted increasing attention in recent years. Using nanotechnology to develop medicines based on glucose metabolic regulation has become a promising strategy. Combining the metabolic therapy of glucose with other therapeutic strategies to achieve better therapeutic effects will be an important future research direction.

### Glutamine and Glutathione Metabolism

Glutamine (Gln) is a nonessential amino acid and an important metabolic fuel that participates in multiple biological processes, including biosynthesis, signal transduction, and protecting cells from oxidative stress (Matés et al., 2019). Gln is absorbed by cells through alanine–serine–cysteine transporter 2 (ASCT2). Glutamine is further converted into glutamate and α-ketoglutarate (α-KG) in mitochondria by glutaminase enzymes and by glutamate dehydrogenase (GDH) or aminotransferases (Jin et al. 2015), respectively. Thus, it can be seen that Gln is an alternative source of carbon elements to replenish the TCA cycle (Masisi et al., 2020). Under hypoxia or mitochondrial dysfunction, α-KG is carboxylated into citrate by isocitrate dehydrogenase. The citrate is exported to cytosol and further transferred into *de novo* fatty acid synthesis or produces another amino acid. In the cytoplasm, glutamine provides an amide (γ-nitrogen) group, which enables nucleotides to be synthesized from scratch. Glutamate produced during this process is further transformed into reduced glutathione (GSH), which plays a key role in protecting cells from oxidative damage and maintaining redox homeostasis (Forman et al., 2009).

Cancer cells exhibit addiction to Gln (Wang et al., 2018). Targeting Gln has become an attractive anti-cancer strategy using nanoplatform-based drug delivery systems. 6-diazo-5-oxo-l-norleucine (DON) is a reactive diazo glutamine analog that binds to multiple enzymes in glutamine metabolism. DON displays anti-tumor activity as a glutamine antagonist in animal tumor models (Lemberg et al., 2018). A therapeutic platform was designed, which combined porous Pt–Pd nanoflowers (Pt–Pd NFs) with DON (Pt–Pd@DON) and was used to enhance electrodynamic immunotherapy (Chen et al., 2022). Under the promotion of DON, the joint functions of the immunogenic cell death (ICD) effect and CD8^+^ T cell infiltration stimulate an anti-cancer immune reaction in immunosuppressive tumors and exert a therapeutic effect. Moreover, inhibiting the activity of key enzymes could not only cut the nutrition supply for tumor cells via blocking of glutaminolysis but also disrupt the intracellular redox homeostasis. The overexpressed GDH1 can promote α-KG generation and is a key regulatory target. A group developed a nanoparticle by inhibiting mitochondrial glutaminolysis for preventing the nutrient supply of tumor cells (Xu et al., 2021). This tumor-targeted theranostic nanoplatform was constructed using the bovine serum albumin (BSA), ferrocene, and GDH1 inhibitor purpurin. BSA provides long circulation and well biocompatibility, and the ferrocene-triggered Fenton reaction provides effective chemodynamic therapy (CDT).

The glutamate-derived GSH is the main redox buffer in cancer cells. Therefore, consuming GSH is considered to be an effective solution for fighting cancer. Numerous nanomedicines, by delivering GSH-depleting agents, have achieved decent therapeutic effects. Chen et al. developed a CD44-specific targeting nanoreactor (AM-L@NBS) that can exhaust the intracellular GSH and cause apoptosis in cancer cells (Shi et al., 2021). The maleimide on the AM-L@NBS interacts with GSH via Michael addition, thereby resulting in the annihilation of GSH and an increase in ROS production, which facilitates the anti-cancer effect. As a reducing substance in cells, GSH can be consumed by reacting with oxidizing agents. General strategies of depleting intracellular GSH mostly are mainly based on the Fenton reaction or Fenton-like reaction. The available GSH-depleting components include various oxidizing agents, such as MnO_2_ (Lin et al., 2018), Cu^2+^ (Xiao et al., 2021), Fe^3+^ (Shen et al., 2020), and Ce^4+^ (Dong et al., 2020). For example, Xiao et al. presented a multifunctional intelligent nanoplatform CuO2@mPDA/DOX-HA (CPPDH), which induced the consumption of GSH and the self-supply of H2O2 (72).

Other glutamine metabolism antagonists (such as ASCT2 antagonist) have also shown antitumor activity in preclinical models (Stine et al., 2021). In a theoretical sense, glutamine metabolic drugs can target glutamine-dependent tumor cells, thereby being applied to different types of cancers, which could be exploited as a “metabolic checkpoint” for tumor immunotherapy (Leone et al., 2019). The related nanomedicine may be one of the development directions in this field.

### Lipid Metabolism and Nucleotide Metabolism

FAs and cholesterol are necessary for cell membranes and other key structures. In addition, lipid metabolism is also related to bioenergy synthesis and signaling molecules needed for proliferation (Röhrig and Schulze, 2016). Dysregulation of lipid metabolism is a prominent metabolic characteristic of cancer cells (Bian et al., 2021). The alterations of lipid metabolism in tumor cells mainly include abnormal upregulation of *de novo* lipid synthesis and FAO [(Carracedo et al., 2013)]. The main substrate for lipid synthesis is cytoplasmic acetyl-CoA: both FAs and cholesterol are synthesized from acetyl-CoA through a series of reactions. Key enzymes involved in acetyl-CoA production, FAs’ biosynthesis, cholesterol biosynthesis, and FAO are key methods targeted to destroy lipid metabolism in cancer treatment (Bian et al., 2021).

Hyperactive acetyl-CoA and FAs production in cancer is mediated by the increase in key enzymes. The main targets commonly used in preclinical and clinical research of drug development include ATP citrate lyase (ACLY), acetyl-CoA carboxylase, and fatty acid synthase (Stine et al., 2022). A study reported that nanomaterials with peroxidase-like activity inhibit tumor growth *in vivo* through an ACLY-dependent rat sarcoma viral oncogene (RAS) signaling mechanism (Wang et al., 2020b). Moreover, the success of therapeutic efficacy of targeting key enzymes supports the potential to deliver counterpart inhibitors through nanoparticles in the future (Wang et al., 2022a). Monoacylglycerol lipase (MGLL), an important enzyme catabolizing lipid that extensively exists in pancreatic cancer cells, plays an important role in triacylglycerol (TG) metabolism. Cao et al. (2022) developed a reduction-responsive poly nanoplatform to deliver MGLL siRNA (siMGLL). This platform can efficiently silence MGLL in cancer cells and lead to the inhibition of free FAs (FFAs) generation and tumor growth. Ferroptosis is a regulatory cell death triggered by lipid peroxidation of membrane unsaturated FAs catalyzed by iron ions (Jiang et al., 2020). It is an attractive target for anti-cancer treatment in nanotechnology (Shan et al., 2020). The design principle of many nanoparticles is based on increasing the lipid peroxidation level of tumor cells by providing exogenous FAs, thereby synergistically inducing iron death (Zhou et al., 2017; Gao et al., 2019a).

The proliferation of tumors depends on *de novo* nucleotide synthesis (pyrimidines and purines). One-carbon (1C) metabolism includes a series of interconnected pathways, providing 1C units (methyl groups) for nucleic acid synthesis (Ducker and Rabinowitz, 2017). Therefore, these pathways contain many promising therapeutic targets for disrupting mRNA synthesis and DNA replication in cancer cells. DNA damage repair pathways are also a common target in clinics for small-molecule inhibitors, chemotherapy, and nanomedicine (Stine et al., 2021). Mut-T homolog 1 (MTH1) is a protein that can inhibit the deoxynucleotide damage in DNA. The effective inhibition of MTH1 of a self-delivery photodynamic synergists nanoparticle could augment DNA damage and promote tumor cell apoptosis (Li et al., 2021c). Many nanoparticles encapsulate inhibitors of DNA damage repair that have been used clinically. For example, the therapeutic effect of BRCA-deficient breast cancer can be improved by encapsulating tarazolpani in bilayer nanoliposomes (Zhang et al., 2019a). In a similar manner, Wang et al. (2020c) designed an amphiphilic peptide nanoparticle encapsulating olaparib and JQ1 to treat non-BRCA mutant pancreatic cancer by inhibiting DNA damage repair pathways. The same idea could be seen in other nanoparticles loaded with doxorubicin to interfere with DNA/RNA synthesis. (Chen et al., 2020; Yang et al., 2021).

## Tumor Microenvironment Metabolism and Targets

The TME is composed of diverse cell populations in a complex matrix, which includes tumor cells, extracellular matrix, immune cells (myeloid and lymphoid lineage), supporting cells (fibroblasts, stromal cells, and endothelial cells), and various other components (Quail and Joyce, 2013; Quail and Joyce, 2017; Hinshaw and Shevde, 2019; Li et al., 2021a). Tumor cells, fibroblasts, or inflammatory cells secret various pro-tumorigenic proteases, cytokines, and growth factors, thereby supporting growth, angiogenesis, and invasion of tumor cells (Quail and Joyce, 2013). Meanwhile, under the attraction of chemokines, immune cells enter and locally proliferate, differentiate, and function in the TME, which includes innate immune cells (macrophages, neutrophils, dendritic cells, innate lymphoid cells, myeloid-derived suppressor cells, and natural killer cells) and adaptive immune cells (T and B cells) (Hinshaw and Shevde, 2019).

For decades, an important limiting factor in the clinical transformation of nanomedicine has been the heterogeneity of tumors. To circumvent this tumor cell heterogeneity, the academic community has shifted attention to leveraging immune cells (Zhang et al., 2020), which are less heterogeneous than tumor cells in the TME [(Trinh and Polyak, 2019)]. On the one hand, immune cells play vital roles in anti-tumor immunity, thereby making targeted immune cell metabolism a promising therapeutic strategy. On the other hand, the behavior of cancer is also regulated by the inherent metabolism of cancer cells and metabolites in local TME [(Augustin et al., 2020)]. Metabolic changes in cancer cells have reshaped the TME and promoted the progression of tumor: glucose, amino acid, and oxygen compete with immune cells, and lactate secretion promotes the formation of immunosuppressive TME (8). For example, tumor cell exerts immunosuppressive functions by inhibiting the infiltration of effector T cells, promoting the regulatory T cell (Tregs) differentiation, and accumulating lactic acid and carbon dioxide (Kouidhi et al., 2017). Meanwhile, the complicated metabolic patterns of noncancer cells within TME also affect the differentiation of its own subsets and increase the immunogenicity of the tumor (Xia et al., 2021). That implies that an essential consideration should be given to the possible beneficial or adverse effects on TME in the future design of metabolic nanodrugs. DRP-104, a glutamine antagonist example that can increase the immune cell response, is a small-molecule metabolic inhibitor undergoing clinical trials (NCT04471415).

Recent research on cancer metabolism has explosively increased but mainly focused on tumor cells. Research on the metabolism of TME is an important direction in the future. The metabolic components and pathways of noncancer cells within TME have also undergone reprogramming and contributed to tumor progression. In this section, we will summarize the alterations of noncancer cells within TME (Figure 2) and metabolic regulation nanoparticles that act on the metabolites of the TME and the surrounding immune or stromal cells (Table 2).

**FIGURE 2:** The metabolites are shaped by noncancer cells within the tumor microenvironment (TME), which have unique metabolic profiles and vulnerabilities. Under hypoxia conditions, the metabolites produced by tumor cells are regulators of noncancer cell function, such as lactate and PGE2. The metabolic pathway alterations of noncancer cells within TME are depicted in different colors (red: upregulation and green: downregulation). These alterations provide a promising direction for the development of nanomedicine: targeting metabolism to improve the TME for cancer treatment.

### Metabolites Within Tumor Microenvironment

The competition and crosstalk of metabolites between different cell types of TME are important determinants of cancer. Tumor vascular abnormalities restrict oxygen exchange and create regions of hypoxia (Fukumura et al., 2018). Metabolic reprogramming of hypoxic cells and disordered blood vessels increases the production and accumulation of immunosuppressive metabolites: lactate, kynurenine, prostaglandin E2 (PGE2), etc. (Chen et al., 2015; Pérez-Tomás and Pérez-Guillén, 2020). Targeting these metabolic features and metabolites, such as hypoxia and low pH, has been a promising strategy in different types of cancer (Bader et al., 2020; DePeaux and Delgoffe, 2021).

Among them, lactate acidifies the TME (pH 6.5–6.8) (Webb et al., 2011) and plays multifaceted roles in local TME, including impairing the immune responses and involving intracellular metabolic crosstalk (Lyssiotis and Kimmelman, 2017; Certo et al., 2021). In detail, accumulation of lactate is deleterious for T cell effector function and anti-tumor response (Fischer et al., 2007). The lactic acid in TME is an active checkpoint for the function of regulatory T cells by promoting PD-1 expression (Kumagai et al., 2022). Lactate also has a critical function in tumor-associated macrophages (TAMs) and myeloid-derived suppressor cells (MDSCs) polarization (Chen et al., 2017b; Zhao et al., 2022). Moreover, cancer cells of normoxia regions consume lactate generated by the hypoxic cancer cells and cancer cancer-associated fibroblasts (CAFs) to fuel the TCA cycle (Lyssiotis and Kimmelman, 2017). One strategy for nanomedicines is to encapsulate lactate oxidase (LOX) and consume lactic acid in the TME by catalyzing its oxidation. A cascade catalytic nanosystem delivers LOX and glycolysis inhibitor with hollow MnO2 (HMnO2) nanoparticles to realize lactic acid exhaustion, which is used for synergistic metabolic therapy of tumors (Gao et al., 2019b). A tannic acid (TA)-Fe (III) coordination complexes-coated perfluorooctyl bromide (PFOB) nanodroplets also load with LOX (PFOB@TA-Fe (III)-LOX, PTFL), which is used for the simultaneous consumption of lactic acid and ATP, and simultaneously generates hydroxyl OH radicals (Tian et al., 2021).

Kynurenine can accumulate in IDO-positive cancers, which is related to the inactivation of effector T cells and promotes immunosuppressive cells (Bader et al., 2020). The kynurenine pathway is controlled by the rate-limiting enzyme indoleamine-2,3-dioxygenase (IDO1) (Platten et al., 2019). IDO1-modulation nanoparticles are always used as an immunometabolism drug to block kynurenine metabolic pathways (Jiang et al., 2021; Liu et al., 2021; Wang et al., 2022b). A work utilizes aza-fused conjugated microporous polymer (aCMP) nanosheets inducing dual-type of ICD and the interference of the IDO pathway in hypoxic tumors (Jiang et al., 2021). Furthermore, cancer cells secret PGE2, thereby directly inactivating T cells. It has been proved that the elimination of PGE2 by inactivation of cyclooxygenase -2 (COX-2) based on nanoparticles could inhibit the growth of tumors (Feng et al., 2022). The group solved the challenge of pharmacokinetic differences and the spatial barrier that PD-1/PD-L1 interaction occurred outside the cell while COX-2 was located intracellularly: this intelligent nanoparticle could release celecoxib (COX-2 inhibitor) in cells in response to the elevated GSH concentration inside tumor cells.

Acidic/hypoxia TME has a close relationship with immune suppression, and it is important for nanodrug development (Watson et al., 2021). These physiological characteristics of TME make it convenient to design the programmed release nanoparticles. Furthermore, taking advantage of the metabolic characteristics of TME, nanomedicines have a better immune response and therapeutic improvement (Huang et al., 2019; Xing et al., 2019; Wang et al., 2022b). For example, a carbonate (CaCO3) nanoparticle was developed to encapsulate 4-phenylimidazole (4PI), thereby inhibiting IDO1 from constructing an acidic pH-activatable nanomedicine, which reinforces the immunity and treatment outcome of radiotherapy (Huang et al., 2019). A multifunctional nanoplatform was constructed using fluorinated polymer nanoparticles and encapsulated with IDO1 inhibitor (NLG919) for pH-responsive metabolic therapy (Xing et al., 2019). This nanoparticle alleviated the hypoxia situation of the TME and improved the therapeutic efficiency.

Cancer cells can also produce various other immunosuppressant metabolites (Stine et al., 2022), such as adenosine and 2-hydroxyglutarateand methylthioadenosine, which offer developers more choice in this field. It can be seen as an optimization direction of nanomedicines that can specifically be activated by simultaneously targeting metabolites and reinvigorating the antitumor immune response.

### T Cell Metabolism in the Tumor Microenvironment

The heterogeneity of antitumor immunity depends, to a great extent, on the diversity and composition of T cells in TME [(Woolaver et al., 2021)]. Existing cognition has identified that metabolism is an important regulatory factor for T cell biological behavior and function (Klein Geltink et al., 2018). Extensive efforts have been made to explore metabolic changes in effector T cells and Treg cells in the TME, which have important therapeutic significance for the development of nanomedicines.

Unlike quiescence status, effector T cells (Teff) activation generally adopts an anabolic metabolism phenotype, which mainly depends on glycolysis and glutaminolysis to rapidly increase the energy supply to achieve proliferation and effector functions (Sharabi and Tsokos, 2020). Activated T cells also upregulate the lipid synthesis, PPP, and one-carbon metabolism pathways, which play important roles in membrane synthesis, nucleotide biosynthesis, and cellular redox balance (Wei et al., 2021). The biochemical intermediates of metabolic reprogramming are essential for the biosynthesis process (nucleotides, amino acids, and lipids) (MacIver et al., 2013). Competitive consumption of glucose by tumor cells restricts the cytotoxicity of Teff (Chang et al., 2015). Therefore, metabolic reprogramming of Teff cells may be a feasible strategy. Nanotechnology has already made some achievements in this field. For instance, it has been reported that promoting fatty acid metabolism could activate T cells and fight against tumor cells (Zhang et al., 2017). A study (Kim et al., 2021) designed a T cell-targeting nanoparticle (aCD3/F/AN) encapsulating the lipid metabolism-activating drug, fenofibrate, which can further activate fatty acid metabolism and restore mitochondrial functions. aCD3/F/AN can specifically target T cells by modifying the surface of nanoparticles with an anti-CD3e f (ab′)2 fragment and exerting an effector-killing effect against tumor cells. Another example is that the function of T cells is affected by the metabolism of cholesterol. Avasimibe (Ava), an inhibitor of the cholesterol-esterification enzyme acetyl-CoA acetyltransferase 1 (ACAT1), potentiates the antitumor response of CD8 (+) T cells by regulating cholesterol metabolism (Yang et al., 2016). Nanomaterials can also be attached to T cells in a strategy known as “backpacking” to carry liposomal Ava in order to enhance solid tumor immunotherapy (Hao et al., 2020). In addition to specific targets within T cells, the metabolism regulation of tumor cells can improve T cell-associated immunity. The knockdown of lactate dehydrogenase A (LDHA) in tumor cells by RNAi nanoparticles, pyruvate metabolism, is reprogrammed to increase CD8^+^ T and NK cells infiltration (Zhang et al., 2019b).

In contrast, regulatory T cells (Treg) cells are essential for tumoral immunosuppression and mainly rely on OXPHOS and FAO for survival (Yu et al., 2018). The specific metabolic mechanisms involving differentiation and maintenance remain unclear. Recent advances in Treg metabolism shed new light on further understanding of the balance of metabolism in TME. For instance, increased uptake of lactic acid can induce Treg cells to express PD-1, and MCT1 is an important metabolic checkpoint in this process (Kumagai et al., 2022). In addition, it is reported that lipid modifications mediated by bidirectional metabolic signaling are important for differentiation and maintenance, which provides a potential target for Treg cell regulation (Su et al., 2020). Some developed drugs are also found to be involved in the metabolic process of Treg cells. Imatinib, a BCR-ABL kinase inhibitor, induces apoptosis of Treg by downregulating the expression of IDO [(Beckermann et al., 2017)]. A hybrid nanoparticle enhances the effect of imatinib in downregulating Treg cell suppression for targeting and modulating Treg cell function in the TME (Ou et al., 2018).

### Other Adjacent Cells’ Metabolism in the Tumor Microenvironment

Besides T cells, there are many kinds of cells in TME, such as dendritic cells (DCs), CAFs, TAMs, and MDSCs (Hinshaw and Shevde, 2019). Among them, CAFs account for the largest proportion of stroma. The function of TAMs and MDSCs is to act as an inhibitor for anti-cancer immunity and to promote tumor progression and metastasis (Gabrilovich, 2017). These cells sense the change in TME and respond by reprogramming the metabolic pathways to maintain the function of suppressive and pro-tumorigenic. Recent progress in these adjacent cells based on metabolic features not only deepens our insight into their metabolic phenotype but also brings nanotargeting therapies onto the agenda.

The promoting functions that CAFs exert on cancer development make them tempting therapeutic targets. Some progress in nanomedicine has been made in this field. For example, it has been reported that the activation of CAFs enhances the delivery of doxorubicin in graphene-based nanosheets (Kim et al., 2017). CAFs were recently reported to undergo upregulated pathways of glycolysis and glutamine and FAs synthesis (Yan et al., 2018a; Becker et al., 2020; Gong et al., 2020). As opposed to tumor cells, CAFs exhibit a catabolism phenotype, which is characterized by the shift in glucose metabolism, referred to as the reverse “Warburg effect” [(Martinez-Outschoorn et al., 2011)]. The self-metabolic reprogramming of CAFs provides fuel (lactate, fatty acid, and amino acids) for biosynthesis in cancer cells (Li et al., 2021d).

TAMs and their influence on the metabolic profile of the TME constitute promising targets for the development of novel anti-cancer nanoagents. Glucose metabolism is vital for the polarization and anti/pro-tumoral function of TAM (Leone and Powell, 2020; O'Neill and Artyomov, 2019). Different macrophages get energy in different ways: M1 macrophages get energy through glycolysis with a fast energy supply and M2 macrophages obtained by OXPHOS (143) and account for the main subgroup in TME. Contrary to the M1 subtype, M2-TAMs exhibit elevated OXPHOS, glutamine, and fatty acid consumption (Vitale et al., 2019). While M1-TAM has a high glycolytic rate, fatty acid synthesis, and increased PPP (Rabold et al., 2017).

The metabolic environment change can affect the polarization and function of TAM subsets. For instance, a CaCO3-based nanoparticle scavenging of H+ provides a simple approach to promoting M1-like macrophage polarization (Chen et al., 2019). Besides, in the model of atherosclerosis (van Leent et al., 2021), nanobiologics that inhibit the genes involved in the energy metabolism of macrophages suggest that the metabolic reprogramming shaped by nanotechnology can phenotypically and functionally affect TAM’s behavior.

The immunosuppressive functions of MDSCs are characterized by the increased accumulation of lipids and FAO. In their differentiation and activation, MDSCs exhibit an increase in glycolysis, glutaminolysis, and the PPP during a decrease in OXPHOS [(Veglia et al., 2021)]. Inhibiting the proliferation of MDSCs may be a safe and effective strategy for cancer intervention. A previous study has reported that the nanosized pseudoneutrophil cytokine sponges (pCSs) can disrupt the expansion and trafficking of MDSCs to improve the cancer immunotherapy effect (Li et al., 2020b).

## Challenge and Outlook

The development of the understanding of tumor metabolism provides a perspective; that is, metabolic molecules that determine the fate of single cells can be used to determine the life and death of an individual (Cassidy et al., 2019). Since the milestone of the cancer metabolism that the FDA approved inhibitors of mutant enzymes for AML [(Pirozzi and Yan, 2021)], metabolic anti-cancer therapy has aroused extensive interest for its potential for cancer treatment. This blossoming field has made some significant progress, but there are still some obstacles to realizing the therapeutic potential of nanomedicines in the clinic.

### Metabolic Nanomedicine Superiority

The traditional strategy of metabolic-targeting drugs has some limitations, such as insufficient drug distribution specificity and systemic toxicity (Yan et al., 2018b; He et al., 2020). However, nanotechnology has greatly broken through these limitations because of its selective targeting, increased drug payload and controlled release, and good biocompatibility (Kim et al., 2010; Niu et al., 2018; He et al., 2019). The application of nanocarriers in metabolic treatment strategy can enhance the accumulation of cargo drugs in local TME, increase the tolerated dose, and promote the curative effect.

Benefiting from elaborate nanotechnology, various metabolic-targeting drugs/molecules encapsulated with nanoparticles show remarkable targeting and anti-cancer abilities (He et al., 2018a; Yan et al., 2020b; Yan et al., 2021b). This superiority is partly due to the well-known enhanced permeability and retention (EPR) (Maeda et al., 2000) and partly because of the elaborate design of nanoparticles to realize better-targeting tropism (He et al., 2022; Li et al., 2022; Ma et al., 2022). Examples of the above research show that nanoparticles can load specific therapeutic molecules (Liang et al., 2021), and change their physical properties (Cui et al., 2021) to achieve precise delivery or specific response. The reasonable design of nanocarriers makes combined medications achieve the optimal synergistic effect (He et al., 2018b; Bian et al., 2018; Ma et al., 2019), which can realize not only dual-pathway targeting but also avoid systemic toxicity.

### Heterogeneity of Metabolism

The heterogeneity of tumors limits the clinical transformation of anti-tumor nanomedicines. The composition of TME is different among the different cancer types. The phenotype of the TME is constantly changing: stromal cells, the composition of growth factors, blood vessels, and immune cells are all in a dynamic state of change (Junttila and de Sauvage, 2013). Corresponding to the phenotype, solid tumors also showed the characterization of significant metabolic heterogeneity (Li and Simon, 2020). Tumor cells from different sources have different characteristics of metabolic gene expression (Xiao et al., 2019). The metabolism in different subtypes of the same tumor is different (Parida et al., 2022). Different regions of the same tumor also exhibit distinct metabolic profiles (Li and Simon, 2020). The metabolic properties and preferences also change during cancer progression (Schug et al., 2016). Above all, tumor cells will adapt to different metabolic modes according to the concentration of external nutrients and different stress conditions (Xia et al., 2021). In other words, cells in different situations and stages will employ different signaling pathways involved in metabolic processes to meet different demands for biological energy and biosynthesis. Therefore, a key consideration is drug specificity. One of the main challenges for active sites is the ubiquity of hydrophobic pockets of metabolizing enzymes (Stine et al., 2022). It is also notable that metabolic plasticity will also result in the impairment of precision-targeted effect (Martínez-Reyes and Chandel, 2021). Many nanoparticle-based drug delivery systems have become suitable carriers to overcome the targeting limitations of traditional drug preparations (Peer et al., 2007; Lim et al., 2019). However, considering the established controversial EPR effect (Ojha et al., 2017) and the limited therapeutic ability of nanomedicines in clinical trials (Wilhelm et al., 2016), tailoring the properties of nanomedicines to increase the target efficiency is still a challenging future direction. Synergistic metabolic therapy that acts on two or more metabolic pathways simultaneously is a way of solving metabolic plasticity (Gao et al., 2019b; Liu et al., 2021). At the same time, dividing patients into different molecular and metabolic subtypes is a clinical method suitable for future personalized treatments.

As the heterogeneity of cancer increases the difficulty of anti-cancer treatment, cancer stem cells (CSCs) provide a possible way to solve this problem (Chen et al., 2021). CSCs-targeting nanomedicine has already become an important research direction and therapeutic target in the development of tumor drugs (Hassani Najafabadi et al., 2020; Zhu et al., 2022). At the metabolic level, CSCs have highly elevated methionine cycle activity and transmethylation rate, which may provide a potential strategy for targeting CSCs (Wang et al., 2019).

### Biosafety and Therapeutic Efficacy

The biological safety of nanoparticles is the premise for clinical application. Targeting metabolism is expected to act on the same enzyme in cancer cells, which may cause toxicity to normal cells (Stine et al., 2022). In particular, current metabolic nanomedicines are effective and safe in animal models, but it is still unknown whether the real effects can be manifested clinically. Therefore, in the long run, the safety profiles of metabolic nanomedicines should be systemically explored, especially in combination with immunotherapy and other agents. In addition, the plasticity and complexity of metabolic networks may result in drug resistance: inhibition of a single metabolic step may cause the replenishment of other pathways (Schug et al., 2016). Compared with the single drug targeting metabolism, the current nanomedicine metabolic strategy mostly adopts combination therapy or blocks multiple pathways (Table 1). The ideal future direction of nanoparticle development is killing cancer cells and synchronously enhancing other strategies, especially those beneficial to immunotherapy. The development of nanotechnology has provided a multifunctional platform for carrying two or more drugs, which provides a broad prospect for the combination treatment of cancer.

In the future, efforts should be made to optimize the characteristics of nanodrugs, such as the material composition, structure, and physical and chemical parameters, to achieve ideal targeted drug delivery, best curative effect, and minimum toxicity.

### Perspective and Conclusion

Metabolism is an active and revolutionary field in oncology, which may be a new checkpoint for anti-cancer treatment (Oh et al., 2021). However, there are still many undetermined issues needing further exploration: 1) distinct cell types have divergent metabolism, but we cannot determine whether the metabolite signals detected are coming from the cancer cells or other cells present within the TME and 2) the metabolic phenotype of many cell types within the TME still needs further investigation. For example, the upregulated aerobic glycolysis is the main pattern of the glucose metabolism of antitumor Teff (Leone and Powell, 2020). That raises the question of whether the activity of Teff will be impaired when we inhibit glucose metabolism in malignant cells. Further, how the metabolism of other cells will be affected when we target a specific metabolic pathway in a specific cell. It is essential to further evaluate the nutritional competition and metabolic interference between neighboring cells and malignant cells. For example, it has long been believed that there is competition between cancer cells and immune cells for metabolic nutrients, such as glucose. But a recent study (Reinfeld et al., 2021) shows that the main culprit of intratumoral glucose consumption by tumors is not cancer cells but immune cells, such as myeloid cells in TME. A recent study reported that the increase in obesity is related to tumor growth and mortality (Turbitt et al., 2019), thereby implying that systemic metabolism is critical for treatment (Lien and Vander Heiden, 2019). Future research needs to determine the mechanism of linking the systemic metabolic state with anti-tumor immunity and use these insights to improve cancer treatment with nanodrugs. Besides, other systemic metabolic factors also play a key role in an anti-cancer immune response. It is worth mentioning that gut microbiota has shown the ability to improve immunotherapy in various preclinical or clinical trials of various cancers (Chaput et al., 2017; Matson et al., 2018; Routy et al., 2018). In addition, some studies have confirmed that antibiotics have negative effects on immunotherapy, thereby indicating that intestinal factors may indirectly affect systemic immune function and anti-tumor immune reaction (Derosa et al., 2018). The underlying mechanism of this connection is attributed to intestinal microbial metabolites (mainly short-chain FAs) (Li et al., 2017). Such systemic metabolism should also be taken into account in the development of nanomedicines.

This review summarizes the latest research progress on nanomedicines in cancer metabolism. This progress includes targeting the metabolic programs of cancer cells and the metabolism of TME. Targeting metabolic pathways is a new field that brings brand-new inspiration for developing anti-cancer nanomedicine. However, it will be a new challenge for the development of nanomedicine to improve anti-cancer immunity while destroying the metabolism of tumor cells.
